The article "SLC41A3 Exhibits as a Carcinoma Biomarker and Promoter in Liver Hepatocellular Carcinoma" was published in 2021. Journal: Comput Math Methods Med.

# SLC41A3 Exhibits as a Carcinoma Biomarker and Promoter in Liver Hepatocellular Carcinoma

**DOI:** 10.1155/2021/8556888

**Published:** 2021-11-15

**Authors:** Qimeng Chang, Yayun Xu, Jianfa Wang, Hui Jing, Longhua Rao, Weiguo Tang, Ziping Zhang, Xubo Wu

**Affiliations:** ^1^Department of Hepatobiliary and Pancreatic Surgery, Minhang Hospital, Fudan University, Shanghai 201199, China; ^2^Institute of Fudan-Minhang Academic Health System, Minhang Hospital, Fudan University, Shanghai 201199, China

## Abstract

Liver Hepatocellular Carcinoma (LIHC) is the fifth widely occurred carcinoma, which is thought to be the second primary contributor of carcinoma-associated death. There are almost 788,000 death tolls worldwide. Solute carrier family 41 member 3 (SLC41A3) is a member of solute carrier family 41, and it is the key point of numerous researches. Our research attempted to explore the links between SLC41A3 and LIHC through public databases. Higher expression of SLC41A3 displayed an intimate association with higher pathological stages and poorer prognosis. GO and KEGG analysis revealed the possible regulatory pathways of SLC41A3. Additionally, we carried out cell functional experiments to determine the expression of SLC41A3 in the cell lines of LIHC, as well as the effects of its silence on cell proliferation, migration, and invasion. Our data showed that SLC41A3 was greatly increased in the cell lines of LIHC. Moreover, silencing SLC41A3 impeded LIHC cell proliferation, migration, and invasion *in vitro*. Collectively, our study demonstrated that highly expressed SLC41A3 was a probable indication of LIHC occurrence, and SLC41A3 could be regarded as a prospective target in the treatment of LIHC.

## 1. Introduction

Among the five commonly occurred carcinomas, Liver Hepatocellular Carcinoma (LIHC) is the second main inducer of carcinoma-associated deaths, reaching 788,000 death tolls worldwide [1–3]. Despite that great improvement has been achieved in early diagnosis and multidisciplinary carcinoma management, a large number of LIHC cases are diagnosed as advanced stage once detected due to the atypical symptoms of early LIHC [4, 5]. Furthermore, LIHC is a highly aggressive and complicated neoplasm disease [6, 7]. The postoperative recurrence ratio is as high as 70% [8]. Herein, setting up an efficacious prognostic model to identify patients with a high risk of recurrence and metastasis is pretty important and urgent. To well understand the probable therapeutic targets and indicators of LIHC will be beneficial for improving the survival ratio in LIHC patients.

Solute carrier family 41 member 3 (SLC41A3) is a member of solute carrier family 41 exhibiting an association with the bacterial Mg^2+^ transporter MgtE, as the main focus of many kinds of research [9–11]. For example, as Mastrototaro et al. demonstrated, SLC41A3 was a mitochondrial Mg^2+^ transporter rather than a plasma membrane protein [11]. It has been shown that SLC41A can promote the outflow of Mg^2+^ from mitochondria and probably modulate the homeostasis of energy [12]. So far, few studies explore the relationship existing between carcinomas and SLC41A3.

Here, we conducted bioinformatics analysis and functional assays *in vitro*. We attempted to explore the relationship of SLC41A3 expression with LIHC. Our results implied that SLC41A3 functioned indispensably in LIHC progression.

## 2. Material and Methods

### 2.1. Bioinformatics Analysis of SLC41A3 in LIHC

Here, we applied gene expression profiling interactive analysis (GEPIA; http://gepia.cancer-pku.cn/) to study the differential expressions of three solute carrier family 41 member genes in LIHC tumor tissues and normal tissues, and also, the relationship of gene expression with neoplasm stages and overall survival (OS) in LIHC patients. GEPIA, a web database, supplies a quick and customizable analysis of genes in various carcinomas. Besides, the Kaplan-Meier Plotter database (http://kmplot.com/) was applied to investigate the association of SLC41A3 expression in neoplasm samples with patients' survival. We plotted the Kaplan-Meier OS curve of LIHC patients with available follow-up data. The log-rank test was applied to determine the difference in survival between groups. The enrichment analysis of GO (Gene Ontology) and Kyoto Encyclopedia of Genes and Genomes (KEGG) was conducted utilizing Enrichr which was accessible at http://amp.pharm.mssm.edu/Enrichr.

### 2.2. Cell Culture and Transient Transfection

HCCLM3, Huh7, MHCC97H (LIHC cell lines), and LO2 (liver normal cell) were supplied by the American Type Culture Collection. They were maintained in DMEM (Gibco, Carlsbad, CA, USA) with 10% FBS (Gibco) and 1% streptomycin-penicillin (Gibco) under a 37°C incubator with 5% CO_2_. For transfection, siRNA of SLC41A3 (si-SLC41A3) was synthesized by GenePharma (Shanghai). 100 pmol of siRNA was transfected into cells by Lipofectamine® 2000 (Invitrogen). We conducted the following experiments at 48 h posttransfection. The siRNA sequence was as follows: si-SLC41A3, 5′-GGGTGCTGATGGTCTGTATAGTGAT-3′; si-NC, 5′-UUCUCCGAACGUGUCACGUTT-3′.

### 2.3. Extraction and Quantitation of RNA

Trizol reagent (Invitrogen) was applied to harvest total RNA from LIHC cells. cDNA was obtained from reverse transfection of RNA utilizing the RevertAid First Strand complementary DNA Synthesis Kit (Fermentas). The relative gene expression was calculated by the iQ SYBR Green Supermix PCR kit (Bio-Rad) on Rotor-Gene 3000 system (Corbett Research). Three tests were carried out, respectively, in this part. The primers were as follows: SLC41A3, forward 5′-GATTGGTGCTCGAAAGCTCG-3′, reverse 5′-CGGCGTCAGATACCGACTA-3′; GAPDH, forward 5′-CTGGGCTACACTGAGCACC-3′, reverse 5′-AAGTGGTCGTTGAGGGCAATG-3′. The transcription level was normalized to the level of the housekeeping gene GAPDH. The relative mRNA level was calculated according to the comparative Ct (*ΔΔ*Ct) method [13], where Ct represents the threshold period of each transcript.

### 2.4. Cell Proliferation

1 × 10^3^ of si-NC-or si-SLC41A3-transfected LIHC cells were plated in per well of a 96-well plate. We conducted a CCK-8 (Cell Counting Kit-8, Dojindo) assay to measure the cell proliferation at 24 h, 48 h, and 96 h as instructions depicted. Taken briefly, we added 10 *μ*l of CCK-8 solution into each well and incubated the cell for 3 h at 37°C. The OD at 450 nm wavelength was measured to count the ratio of living cells. We drew and analyzed the proliferation curve over 4 days with GraphPad Prism 7.0.

### 2.5. Transwell Assays

si-NC or si-SLC41A3 was transfected into LIHC cells before Transwell assays. Then, we starved the transfected cells in the DMEM absence of serum for 6-8 h. We utilized Boyden Transwell chambers (Corning Inc.) with 8 *μ*m membrane filters. 5 × 10^4^ of cells in serum without medium were inoculated in the upper chamber. DMEM with 10% FBS was set in the bottom chamber. After 24 h incubation at 37°C, the cells in the lower chamber were fixed with 100% methanol for 10 min and stained with DAPI (Beyotime Institute of Biotechnology, Shanghai, China) for 15 min at indoor temperature. Positive cells at five random fields were photographed under a 100x light microscope Olympus CX41-32C02 (Olympus Corporation). For invasion assays, Matrigel (BD Biosciences) was precoated in the upper chamber for 6-8 h. 5 × 10^4^ of cells were plated in the upper chamber in a medium without serum. Other procedures were similar to migration assay. Each experiment was carried out three times, respectively.

### 2.6. Statistical Analysis

The derived data were analyzed by GraphPad Prism 7.0 (GraphPad Software, Inc.) and SPSS 22.0 Statistics (IBM Corp) and shown as the mean ± SD. The differences existing in two groups or the differences between paired samples were separately assessed by Tukey's test and paired sample *t*-test. Kaplan-Meier curves plus log-rank tests were both employed to investigate the relationship of SLC41A3 expression with OS. The great statistical difference indicated *P* < 0.05.

## 3. Results

### 3.1. SLC41A3 Was Dramatically Increased and Its Expression Was Related to the Carcinoma Stage in LIHC

To investigate the role of three solute carrier family 41 member genes in the development of LIHC, we evaluated the links between gene expression and the LIHC stage. In the light of the differential expression analysis from the GEPIA database, SLC41A3 was greatly increased in the neoplasm tissues of LIHC than normal tissues (Figure 1(c)). Nevertheless, there was no obvious alteration of SLC41A1 and SLC41A2 expression existing in neoplasm tissues and normal tissues (Figures 1(a) and 1(b)). We assessed the relationship of three gene expressions with LIHC pathological stage from the GEPIA database. It was found that expressed SLC41A1 and SLC41A3 displayed a significant association with the pathological stage of patients (Figure 2(a), *P* = 0.0158 and Figure 2(c), *P* = 0.0176), whereas SLC41A2 expression was not related to patients' pathological stage (Figure 2(b), *P* = 0.0165). Taken together, the expression of SLC41A3 was significantly heightened and exhibited an association with the carcinoma stage in LIHC.

### 3.2. SLC41A3 Was Significantly Related to LIHC Patients' Prognosis

Survival analysis of three solute carrier family 41 genes on the basis of the GEPIA database revealed that highly expressed SLC41A1 and SLC41A3 forecasted poorly prognostic status, but highly expressed SLC41A2 presented a well prognostic outcome (Figures 3(a)–3(c)). Since only SLC41A3 was significantly differentially expressed between LIHC tumor and normal tissues, we further investigated the prognosis of SLC41A3 in LIHC based on the Kaplan-Meier Plotter database. The results confirmed that high SLC41A3 expression in LIHC was significantly associated with poor prognosis (Figure 3(d)).

### 3.3. SLC41A3 Participated in Various Important Biological Processes and Pathways

To elucidate how SLC41A3 participates in human tumor pathogenesis, enriched GO biological process terms and KEGG pathway of SLC41A3 coexpression genes were retrieved from the Enrichr database. The main enriched GO terms in t1he biological process included RNA processing, RNA splicing, and endosomal transport (Figure 4(a)); the mainly enriched GO terms in cellular component were nuclear body, nuclear chromosome part, nuclear speck, and so on (Figure 4(b)); the mainly enriched GO terms in molecular function contained RNA binding, transcription coactivator activity, cadherin binding, and so on (Figure 4(c)). In addition, the top 10 enriched KEGG pathways were spliceosome, endocytosis, ubiquitin-mediated proteolysis, RNA transport, bacterial invasion of epithelial cells, proteasome, Salmonella infection, N-glycan biosynthesis, mRNA surveillance pathway, and shigellosis (Figure 4(d)). These data demonstrated that SLC41A3 participated in various biological processes and pathways especially related to RNA.

### 3.4. *In Vitro* Experimental Results of SLC41A3 in LIHC Cells

To further study SLC41A3 expression in LIHC, we also analyzed SLC41A3 expression in LIHC cell lines by qRT-PCR. The data revealed that SLC41A3 expression was upregulated in LIHC cells and the result was the same as what we found in the GEPIA database (Figure 5(a)). In addition, we discovered that SLC41A3 had the highest expression in HCCLM3 cells, compared with normal others. Thus, it was selected for CCK-8 and Transwell assays.

Next, we knocked down SLC41A3 in HCCLM3 cells by siRNAs (Figure 5(b)). CCK-8 results showed that si-SLC41A3 could certainly weaken cell proliferation rate (Figure 5(c)). Transwell assays also demonstrated that ablating SLC41A3 dramatically weakened LIHC cell migration and invasion abilities of the cells (Figures 5(d) and 5(e)).

## 4. Discussion

Liver carcinoma is also named by hepatic carcinoma and primary hepatic carcinoma. The generally occurred liver carcinoma, accounting for about 75% amid all primary liver carcinomas, is LIHC [14, 15]. LIHC is a malignant neoplasm formed by liver cells, called hepatocytes [16]. LIHC is not sensitive to chemotherapy and radiotherapy [17]. Common treatment methods include surgical resection, liver transplantation, vascular intervention, and radiofrequency ablation [18–22]. Until now, the precise mechanism in LIHC has not been clarified. Further studies need to be conducted.

SLC41A3 is abbreviated from solute carrier family 41 member 3, also called SLC41A1-L2 [23]. It is ubiquitously expressed in the testis, ovary, and 25 other human tissues [24]. The 41^st^ family of solute carriers (SLC41) consists of three members A1, A2, and A3, distantly homologous to bacterial Mg^2+^ channel MgtE [11, 25, 26]. SLC41A1 has recently been characterized as a Na^+^/Mg^2+^ exchanger [12, 25, 27, 28]. It is not well understood that the definite functions of SLC41A2 and SLC41A3, even though they are reported to be involved in Mg^2+^ transport in human cells. Currently, studies on SLC41A3 are few. Herein, our study is aimed at exploring what function SLC41A3 has in cancers. In the present study, we identified that among solute carrier family 41, only SLC41A3 significantly upregulated in LIHC through mining the GEPIA database, the expression of SLC41A3 was positively correlated with the pathological stage of LIHC patients, and higher expression of SLC41A3 was dramatically linked to the shorter overall survival of LIHC patients. These data indicated that SLC41A3 was a LIHC-specific gene and perhaps emerged as a pivotal factor in LIHC occurrence and development.

Additionally, to investigate the biological processes and pathways of SLC41A3 that participated in LIHC, we performed GO and KEGG enrichment analysis of genes coexpressed with SLC41A3. The results revealed that these coexpression genes took part in multiple pathways of RNA-related, containing RNA processing, RNA splicing, RNA transport, RNA binding, and others. It is worth noting that more and more large-scale genome studies have discovered that RNA processing is dysregulated in carcinoma and functionally promoted tumor initiation and maintenance [29]. Therefore, we hypothesized that SLC41A3 might promote the tumorigenesis and progression of LIHC through altered RNA processing.

Finally, our data confirmed that SLC41A3 expression in neoplasm cells of LIHC was significantly increased by qRT-PCR assay. We conducted *in vitro* knockdown experiments, and the data revealed that reducing SLC41A3 impaired LIHC cell proliferation, migration, and invasion. Our results suggested that SLC41A3 might serve as an oncogene in LIHC.

This study has some limitations. First, the expression and protein levels of SLC41A3 should be detected in clinical samples from LIHC patients. Secondly, the function of SLC41A3 should be further verified *in vivo* through animal model tests. In future studies, we will collect more clinical samples from LIHC patients to detect the expression and protein levels of SLC41A3. We will conduct *in vivo* experiments to further analyze the function of SLC41A3.

## 5. Conclusion

In summary, this research firstly revealed the relationship between SLC41A3 and LIHC. After bioinformatics analysis and functional assays, SLC41A3 was increased in LIHC tissues and associated with pathological stages and survival rate in LIHC patients. Silencing SLC41A3 could inhibit cell proliferation, invasion, and migration. Taken together, SLC41A3 functions as an oncogene in LIHC, and it may provide a new perspective for LIHC diagnosis and treatment.

## Figures and Tables

**Figure 1:** Differential expression of solute carrier family 41 family genes in LIHC using the GEPIA database. (a) The expression of SLC41A1 in the neoplasm tissues of LIHC. (b) The expression of SLC41A2 in the neoplasm tissues of LIHC. (c) Dramatical higher expression of SLC41A3 was in LIHC tumor tissues compared to normal tissues. ^∗^*P* < 0.05.

**Figure 2:** Assessment of the relationship between solute carrier family 41 family gene expression and pathological cancer stage in LIHC patients using the GEPIA database. (a) Highly expressed SLC41A1 exhibited a significant relationship with high pathological carcinoma stage. (b) The relationship between the expression of SLC41A2 and pathological carcinoma stage. (c) Highly expressed SLC41A3 displayed an obvious association with high pathological carcinoma stage.

**Figure 3:** Association between the expression level of solute carrier family 41 family genes and prognosis in patients with LIHC. (a) Highly expressed SLC41A1 presented an obvious association with shorter OS of LIHC patients utilizing the GEPIA database. (b) Lowly expressed SLC41A2 had a significant association with shorter OS of LIHC patients using the GEPIA database. (c) Highly expressed SLC41A3 displayed an obvious relationship with shorter OS of LIHC patients using the GEPIA database. (d) Highly expressed SLC41A3 was greatly related to shorter OS of LIHC patients using the Kaplan-Meier Plotter database.

**Figure 4:** Enrichment analysis of SLC41A3-coexpression genes in LIHC. (a) To identify GO biological process terms of SLC41A3 involvement. (b) To identify GO cellular component terms of SLC41A3 involvement. (c) To identify GO molecular function terms of SLC41A3 involvement. (d) To identify KEGG pathways of SLC41A3 involvement.

**Figure 5:** *In vitro* experimental results of SLC41A3 in LIHC cells. (a) SLC41A3 mRNA expression was higher in LIHC cell lines than normal liver cells. (b) SLC41A3 was silenced by siRNA in HCCLM3 cells. (c) Cell proliferation in LIHC cells transfected with si-SLC41A3. (d, e) Cell invasion and migration abilities in LIHC cells transfected with si-SLC41A3. ^∗^*P* < 0.05 and ^∗∗^*P* < 0.01.

## Data Availability

The datasets used and/or analyzed during the current study are available from the corresponding authors on reasonable request.

## Abbreviations

LIHC: Liver hepatocellular carcinoma
SLC41A3: Solute carrier family 41 member 3
GEPIA: Gene expression profiling interactive analysis
OS: Overall survival
GO: Gene Ontology
KEGG: Kyoto Encyclopedia of Genes and Genomes
SLC41: The 41^st^ family of solute carriers.
